The article "A Treatment to Cure Diabetes Using Plant-Based Drug Discovery" was published in 2022. Journal: Evid Based Complement Alternat Med.

# A Treatment to Cure Diabetes Using Plant-Based Drug Discovery

**DOI:** 10.1155/2022/8621665

**Published:** 2022-05-09

**Authors:** Sumalatha Mahankali, Jagadish Kalava, Yugandhar Garapati, Bullarao Domathoti, Venkata rao Maddumala, Venkatesa Prabhu Sundramurty

**Affiliations:** ^1^Department of Mechanical Engineering, Velagapudi Ramakrishna Siddhartha Engineering College, Vijayawada, Andhra Pradesh 520007, India; ^2^Deaprtment of CSE, Dr.A. P. J. Abdul Kalam University, Indor, India; ^3^Department of CSE, GITAM Deemed to be University, Hyderabad, India; ^4^Department of CSE, Shree Institute of Technical Education, Tirupati, Andhra Pradesh 517501, India; ^5^Department of CSE, Vignan's Nirula Institute of Technology and Science for Women, Guntur, Andhra Pradesh, India; ^6^Center of Excellence for Bioprocess and Biotechnology, Department of Chemical Engineering, College of Biological and Chemical Engineering, Addis Ababa Sciecne and Technology University, Addis Ababa, Ethiopia

## Abstract

The field of peptides and proteins has opened up new doors for plant-based medication development because of analytical breakthroughs. Enzymatic breakdown of plant-specific proteins yields bioactive peptides. These plant-based proteins and peptides, in addition to their in vitro and vivo outcomes for diabetes treatment, are discussed in this study. The secondary metabolites of vegetation can interfere with the extraction, separation, characterization, and commercialization of plant proteins through the pharmaceutical industry. Glucose-lowering diabetic peptides are a hot commodity. For a wide range of illnesses, bioactive peptides from flora can offer up new avenues for the development of cost-effective therapy options.

## 1. Introduction

Biomolecules play an important role in the ligand-reason interactions, and their beautiful use in herbal structures triggers the signalling cascade, which is an important aspect of daily life. In dreams, lipids, carbohydrates, and nucleic acids occupy specific receptors. When all of the binding and structural alterations have been completed, a peptide is released as a signal. A contamination can develop if a signal transduction route fails [1, 2]. Those enzymes that break down proteins into bioactive peptides are known as proteolytic reagents. Bioactive peptides, which can contain up to twenty amino acids, do not interact with many proteins because of their short half-life. Affinity for tissue and selectivity, as well as above-average overall performance, are considered favourable conditions [3]. The ability of a peptide's backbone to switch between hydrophobic and hydrophilic states is one example of its structural abilities. Peptide form and herbal pastimes are not inseparable, but it is an essential part of their athletic activities [4]. Regardless of not peptides are bioactive or nutraceutical, they can have a significant impact on an individual's health [5]. Advances in disease prevention and treatment, as well as scientific developments in lifestyle, metabolic, and immunological device trends, are all contributing to an increase in human fitness [6].

The article "A Treatment to Cure Diabetes Using Plant-Based Drug Discovery" was published in 2022. Journal: Evid Based Complement Alternat Med.

As with every drug, each peptide and protein treatment has its own unique set of benefits and cons when it comes to sports injury rehab. With many advantages, however, they also have significant downsides that make them difficult to compete in today's cutting-edge medication market [7]. The manufacture of protein necessitates a number of stages, many of which are expensive. Because oral protein absorption is limited, a move to parenteral nutrition may be desirable [8]. Between 2018 and 2026, the global peptide therapeutics market is expected to grow at a CAGR of 9.1% (2016). Insulin's use as a recovery peptide accounts for a significant portion of the market. J.B. Collip, along with Frederick Banting and Charles Best, became the first person to successfully isolate insulin from a variety of animal sources, thanks to their combined efforts [9]. The biosynthetic insulin brand Humulin was introduced by Eli Lilly and Company in 1983. Insulin was first derived from animal pancreases by a for-profit enterprise. 88.7% of the insulin market is dominated by Novo Nordisk, Sanofi, and Eli Lilly together. Some 22 and two-thirds of the top ten antidiabetic medicine businesses owe money to Sanofi's Lantus, a drug manufactured by the company (basal insulin). Lantus had a revenue of $6.057 billion in 2016. The year 2017 saw the release of Dezzani [10, 11]. While the FDA classifies small molecules and peptides as “New Chemical Entities,” proteins used to treat a wide range of diseases are referred to as “New Biological Entities” (NBEs).

Therapeutic peptides can be used to treat a wide range of medical conditions, including cancer, diabetes, and obesity (Figure 1). When it comes to treating type 2 diabetes, Novo Nordisk's liraglutide (Victoza) has been the top-selling peptide medical medicine in recent years [13], [14]. Glatiramer acetate, a Teva-developed immunomodulator, is used to reduce the symptoms and signs and symptoms of patients with multiple sclerosis [15]. Abbott's leuprolide (Lupron), a hormone responsive therapy, is utilised in the treatment of most cancers and estrogen-based diseases [16]. In the treatment of breast and prostate tumours, the gonadotropin-liberating hormone agonist Zoladex is synthesised by Astra Zeneca and reduces the release of sex hormones [17]. Companies like Amgen, Eli Lilly, Roche, and Pfizer are also researching peptide or protein-based therapies in order to shorten the market advantage for treatment of more advanced problems [13].

The article "A Treatment to Cure Diabetes Using Plant-Based Drug Discovery" was published in 2022. Journal: Evid Based Complement Alternat Med.

It has become more difficult to analyse and purify these compounds, thanks to new analytical systems, cutting-edge purification techniques, and in vitro tests. However, there has been a lot of interest in the use of plant secondary metabolites, which contain small molecules, to transport new capsules to combat disease spread [18].

The discovery of primary metabolites, proteins, and peptides derived from plants has given rise to a new type of examination challenge as shown in Figure 2 [19]. With peptide-based treatments for diabetes becoming more common, the challenges of creating peptide-based medicines and the potential of peptides as healing treatments were also discussed.

Has the potential to totally reverse the diabetes. Oral hypoglycemic medications are commonly used to manage type 2 diabetes. One of the most commonly prescribed medications is metformin, which is supplemented by hypoglycemic agents from a wide range of classes as given in Table 1 [20]. These include thiazolidinediones, alpha-glutamyl transferases, sulphonylureas, and DPP-IV and SGLT-2 inhibitors. Hypoglycemia, fatigue, diarrhoea, and anaemia risk are all associated with these therapies. As these side effects compound over time, they put additional strain on visceral organs such as the heart and lungs, which are already the most commonly concerned devices [21].

Several sources were employed to synthesize exenatide, which was generated from the peptide exendin-4 first obtained from the Gila monster (*Heloderma suspectum*) [22]. Despite their structural similarity to GLP-1, liraglutide and semaglutide have a longer half-life and are not destroyed by DPP-IV [23]. Recombinant DNA technology has made it possible to generate large quantities of these peptides. Synthetic or recombinantly produced peptides are more expensive than tiny molecules, making them out of reach for the general people. Peptide-based pharmaceuticals and herbal-based fitness items have grown increasingly popular [24]. Bioactive peptides derived from animal proteins have been the subject of numerous clinical studies. Discovery of useful leads from plants to improve diabetic patient care is made possible by researchers' excursions into bioactive peptides [25].

### 1.1. Extracts of Plant Peptides with Bioactive Qualities

Bioactive peptides have been overconcentrated in both animal and plant resources [26]. Bioactive peptides are found in animal products such as milk, eggs, meat, and fish that are easily accessible to the general population. There are only a few bioactive peptides that have been isolated from soy, wheat, and other cereals [27]. In animals, overconsumption of protein has been linked to a variety of health issues, including high blood pressure, heart disease, and stroke. Plant-based proteins, on the other hand, do not include fat or produce bad results [28]. As studies have advanced toward a fuller understanding of floral signalling, a new and well defined component in mobile-to-cell communication has emerged: secreted peptides, short RNAs, and transcription factors [29–31]. Plant and animal-derived signalling peptides have now been established to be biosynthesized in a similar manner, despite some of the components of the biosynthesis still being unknown. Early development techniques such as meristem boom, organ loss, cell elongation, cell multiplication, cell differentiation, and invasion defence make extensive use of plant-derived peptides [32]. It has been hypothesised that mediator proteins and peptides evolved in microorganisms and were eventually integrated into higher mediator systems in sophisticated animals at some unknown point in time during evolution [33]. The peptides found in *Spinacia oleracea* L. were among a slew of hormone-like compounds found in flowers. Furthermore, *Lemna gibba* G3, in addition to the ones found in oats and alfalfa as well as the luteinizing *Avena sativa* L. Consider the fact that signalling peptides were discovered a few billion years ago in the fossil record to support this idea [34–37]. Plant proteins, which contain essential amino acids, are an excellent source of nutrition for humans. From leaves to the finished product, there are three types of plant proteins. Seeds (legumes and grains) have a higher protein content than vegetables, and this is reflected in the finished product [38]. Bean seeds from *Vicia faba* and *Lupinus albus* have a protein content of 18–20%, but bean seeds from *Glycine max* and *Lupinus albus* have a protein value of 35–45% (soybean). It is *Lupinus albus* L. (lupin) [39].

The article "A Treatment to Cure Diabetes Using Plant-Based Drug Discovery" was published in 2022. Journal: Evid Based Complement Alternat Med.

Extraction of antibioactivity peptides and hydroysate from plants from bioplants is shown in Figure 3 [40] and benefits are shown in Tables 2 and 3 [20].

### 1.2. Alpha-Glucosidase Inhibitor

Alpha-glucosidase inhibitors compete with enzymes in the intestine that break down nonabsorbable polymers into monosaccharides, resulting in a reduction in absorption. In light of these findings, it was concluded that postprandial plasma glucose levels were significantly lower than they were on a daily basis. Inhibitors of this enzyme may cause beta mobile pressure to decrease (thus decreasing postmeal hyperglycemia) and the production of glucagon-like peptide-1 (GLP-1) to increase (thus increasing insulin secretion) as a result [41, 42]. A reduction in postprandial hyperglycemia in diabetics will raise their risk of developing macrovascular issues, which can be minimised by the administration of insulin throughout the meal [42, 43]. The inclusion of a glycemic opportunity in those items aspires to lessen glucotoxicity while also increasing beta mobile insulin production in the body [41, 44].

Despite the fact that peptides make up the majority of the alpha-glucosidase inhibitors that are commercially available, there are no peptide-based alpha-glucosidase inhibitors available on the market. Peptides derived from flowers have been used in several studies to inhibit the enzyme alpha-glucosidase. An enzyme-blocking peptide derived from hemp seeds contained branched-chain amino acids, hydrophobic amino acids, and essential amino acids, all of which were discovered to be present [45]. The hydrolysate of oat seed proteins is broken down by a protease (alcalase), producing bioactive peptides that have the ability to block the activity of the enzyme alcalase. Additional findings were obtained by an in vivo examination. With an increase in the dosage of oat peptides administered to STZ-induced diabetic mice, the amount of food consumed reduced while insulin production increased. The diabetic mice also demonstrated improved glucose tolerance and glycogenesis [46]. Hydrated peptides produced from the fruit proteins of *Juglans mandshurica* Maxim were selected as antidiabetic agents for clinical trials (walnut). These chemicals work by interfering with the enzyme responsible for sugar breakdown in the body. We discovered that WHPs with molecular weights ranging from 3 to 10 kDa had an inhibitory effect on alpha-glucosidase in vitro, with a 67% inhibitory effect.

Extracellular glucose absorption by insulin-resistant HepG2 cells is significantly increased as a result of the use of this cell type. Several studies have demonstrated that WHPs can lower blood glucose levels by means of lowering insulin manufacture, liver glucokinase interest, and glycogen levels by 64.8% in domestic individuals ordinary [47]. In diabetic version KK mice, researchers discovered enzyme inhibitory properties in proteins derived from the adzuki bean *Vigna angularis* Wild (KK-Ay), which was discovered by chance. In the hours following a meal, the extract helps to reduce postprandial blood sugar levels. In the presence of sucrose challenge conditions, the glucose levels of regular rats and rats treated with streptozocin were 15.6% and 29.9%, respectively. The presence of adzuki bean proteins at a concentration of 10 mg/mL in vitro inhibits the activity of rat intestinal alpha-glucosidase by 60% (2014) [48]. In peptide fractions with molecular weights of 1 kDa and above, a protein-rich extract of *Phaseolus vulgaris* L. (Pinto Durango and Negro 8025) beans was hydrolyzed and ultracentrifuged, and the results revealed that 76% of 0.5% enzyme inhibition was observed [49]. Protein samples from *Phaseolus vulgaris* (black bean) were incubated for hours with an enzyme to substrate ratio (E/S) of 1:20 and a 66.1% inhibition of alcalase hydrolysis, as determined by an enzyme to substrate ratio (E/S) of one to twenty. After in vitro digestion of *Chenopodium quinoa* Willd. (quinoa) protein, LC–MS/MS was used to identify well-known bioactive peptides with amino acid sequences such as IQAEGGLT, DKDYPK, and GEHGSDGNV, among others. At a concentration of 250 million millimetres, it was discovered that enzyme inhibition was 55%, 22%, and 30% at different levels of concentration [50]. Using *Morus alba* L. (mulberry) leaves, researchers discovered that they could produce an oligopeptide with molecular weights ranging between 0.5 and 3 kDa that inhibited enzymes at a concentration of 12.56 g/ml [51]. A protein that is contained within the form of the plant, *Momordica cymbalaria*, is presented by Hook.f. (*Momordica cymbalaria*). In animal studies, it has been demonstrated that inhibiting enzymes responsible for a decrease in glucose production helps to improve the carbohydrate metabolism [52].

The article "A Treatment to Cure Diabetes Using Plant-Based Drug Discovery" was published in 2022. Journal: Evid Based Complement Alternat Med.

### 1.3. Inhibitors of Alpha-Amylase

As part of the process of converting nonabsorbable polysaccharides into absorbable monosaccharides [53], amylase (*α*-1,4-glucan-glucanohydrolase) aids in weight loss by increasing carbohydrate and starch hydrolysis (*α*-1,4 glycosidic linkage) and decreasing fat absorption [54]. Amylase inhibitors lower blood glucose levels after a meal as a result of the fact that they delay the digestion of carbohydrates and the absorption of glucose into the bloodstream [55].

It is possible that pinto beans, despite the fact that they have not been extensively studied, may also have some health benefits. It had been decided to dialyze the hydrolyzed fraction for 1 h at 50°C with an (E/S) ratio of 1 : 10, and the fraction obtained with molecular weight tonnes an awful lot a good deal less than 3 kDa revealed 62% and 3%, respectively. 49% and 5% enzyme inhibition, respectively, were observed during the enzymatic digestion of the pinto bean protein fraction employing protease (Protamex) at pH 6 [56]. Dialysis and bromelain (protease) were thought to be particularly effective at inhibiting enzyme activity. Only one-fourth of 1% is consistent with the previous year [49]. The alpha-amylase inhibitory peptide CSP1, which was derived from cumin seed, lowered alpha-amylase activity by 24.54% points in vitro [57]. It was discovered that *Triticum aestivum* L. (wheat) albumin extract inhibited the enzyme alpha-amylase, resulting in reduced blood glucose levels following a meal as a result. Postprandial glucose levels have been lowered by using 31% of the dose at the same time as using 0% of the dose. For 25 g sample, the answer is zero. 5 g and 100 g of wheat albumin were used and the answer is zero. Although the addition of 5 g wheat albumin had no effect on fasting blood glucose levels, it did have a positive effect on haemoglobin A1c levels, which are a measure of diabetics' metabolic control, in an extended-term manipulation study [58]. It has been determined through research that *Hordeum vulgare* (barley) flour has been submitted to pancreatic hydrolysis and that peptides isolated from the flour have a 57–77% inhibitive impact on the enzyme alpha-amylase. Cucurbitin, a protein found in the seeds of *Cucurbita pepo* L. pumpkins, has been shown to inhibit the hydrolysis of alcalase and pepsin, two enzymes involved in digestion. The C50 value for mulberry oligopeptides has been increased from 12 to 14. It is believed to have the most inhibiting reputation at a concentration of 25 g/ml. Laminar go together with the flow. *Moringa oleifera* (moringa tree) extracts of protein hydrolysates from seeds have been developed. The enzymes trypsin, chymotrypsin, and pepsin-trypsin are utilised for the first two and a half and five hours, respectively. The use of the pepsin-trypsin digested fraction for hydrolysis intervals of 5 h and 5 h, respectively, for alpha-amylase inhibition was validated, with IC50 values of 0.195 and 0.123 g/ml, respectively, confirming the findings of the previous research [59]. The IC50 for alcalase hydrolysate was modified and determined to be 0.149 mg/ml for protein hydrolysate of watermelon seeds received with the useful beneficial resource of enzymes together with pepsin, trypsin, and alcalase [60]. Three different PH values were employed to construct *Theobroma cacao* L. that give up end outcome autolysates: 3.5, 5.2, and 5.3. In vivo tests showed that when the autolysate has emerged at pH 3.5, alpha-amylase inhibition and insulin launch have been maximised and blood glucose stages have been decreased [61]. Quinoa protein fractions reduced alpha-amylase by 6.86% at 250 mg/ml after enzyme hydrolysis of quinoa proteins, according to the results of the experiment [50].

The article "A Treatment to Cure Diabetes Using Plant-Based Drug Discovery" was published in 2022. Journal: Evid Based Complement Alternat Med.

### 1.4. Dipeptidyl Peptide IV Inhibitors

Incretin hormones, such as GLP-1 and GIP, are two of the most significant gut-derived hormones, and their role in controlling blood glucose levels is well-known [62]. Along with the decrease in appetite and insulin release, the level of the hormone glucagon also decreases [63]. The incretin hormone is released at a lower rate in diabetics. These hormones display their herbal consequences as they link with receptors in the colon [64]. A return to normal hormone production or a reduction in hormone breakdown is an aspect of diabetes treatment. GLP-1 is degraded with the help of DPP-IV within minutes of its creation, leaving it without any herbal trends. Inhibition of DPP-IV could be a useful tool in the fight against hyperglycemia. DPP-IV inhibitors enhance GLP-1 postprandial effects by delaying GLP-1 breakdown, which lowers hepatic glucagon era, activates pancreatic beta cells, and raises insulin levels.

With an IC50 cost of 1.450, dipeptides produced from rice bran protein hydrolysate inhibited the DPP-IV enzyme.

13 mg/ml protein was from rice bran [65]. Rice bran protein fractions were defatted and hydrolyzed using Bioprase SP and Umamizyme G in pioneering research. Following dipeptide digestion with Umamizyme G, IC50 was discovered to be 2.3, 0.1 mg/ml [66]. Proteins from *Amaranthus hypochondriacus* L. were employed to make bioactive peptides by simulating gastrointestinal digestion. With an IC50 of 1.1 mg/ml, this peptide fraction has been shown to inhibit enzymes dose-dependently [67]. *Glycine max* L. (soybean), *Lupinus albus*, and Lup 1 protein hydrolysate all included DPP-IV inhibitory peptides. Soy 1 and Lup 1 were inhibitory peptides with IC50 values of 106 and 228 M, respectively [68]. CPGNK and GGGLHK, herbal peptides derived from the protein digestion of not top-notch beans, inhibited enzyme activity with IC50 values of 0.87, 0.02, and 0, respectively. In the neighbourhood, there are 610.10 peptides (Mojica et al., 2017, [69, 70]). Proteins produced from *Phalaris canariensis* L. (Canary) seed inhibited DPP-IV digestion in the gastrointestinal tract by 40% [71]. The IC50 for papain inhibition of quinoa proteins was reported to be 0.88 for 0.05 mg/ml using hydrolysate-papain hydrolysate [72]. Quinoa protein was employed to complete a simulated duodenal digestion, and the IC50 (mg protein/mL) was found to be zero. The amount of protein per millilitre is 840.007 [50].

### 1.5. Transporter Inhibitors for Glucose (GLUT and SGLT)

In order for glucose to pass through the lipid bilayer of the membrane, membrane proteins (glucose transporters) function along the lipid bilayer [20]. Glucose is passively transported by GLUT transporters, which do not require energy to function, but active glucose transport by SGLT transporters necessitates energy. This method results in salt transfer from one location to another, so that glucose can be added to the membrane's route [73, 74]. In the human body, there are at least 12 extraordinary GLUT transporters and 7 remarkable SGLT transporters, all of which may be membrane-elastic protein members. The proximal tubule reabsorbs 90% of the ejected glucose, whereas the distal tubule reabsorbs the remaining 10%.

The article "A Treatment to Cure Diabetes Using Plant-Based Drug Discovery" was published in 2022. Journal: Evid Based Complement Alternat Med.

In response to high blood glucose levels (hyperglycemia), the proximal tubule detects an increase in the expression of a glucose transporter gene [20]. Peptides that specifically target plant glucose transporters have been tested in a limited number of cases to a great effect. Antiglycose transporter inhibitors with amino acid sequences AKSPLF and ATNPLB have been demonstrated to be effective in the treatment of diabetes. After 24 h of therapy with the Caco-2 cellular version, the bioactive peptides examined reduced glucose reabsorption by 21.5%. The oral glucose tolerance test in rats after 50 mg of hydrolyzed protein isolate/kg BW showed a 24.5% reduction in postprandial hyperglycemia (*P* 0.05) (Mojica et al. 2004).

### 1.6. Insulin Replacement Remedy

Insulin regulates the metabolism of a weight loss plan via a series of signalling pathways [22]. In response to insulin, the alpha subunit of the insulin receptor undergoes conformational changes, which activates cytoplasmic tyrosine kinase. As a result, insulin transphosphorylates additional intracellular substrates before activating the insulin receptor. When these outcomes are coupled, they have severe effects on metabolic and mitogenic structures [75]. The activation of tyrosine kinase by insulin mimics has implications for receptor autophosphorylation and downstream insulin signalling. Furthermore, the insulin mimic (vanadate) functions by blocking tyrosine phosphatase from dephosphorylating insulin receptors, reducing insulin sensitivity [76].

According to the radioimmunoassay, spinach and *Lemna gibba* G3 extracts imitate mammalian insulin. According to an in vivo study in extra young rats, a plant insulin-like fibre interacts with insulin receptors on IM-9 lymphocytes and supplements glucose oxidation and lipogenesis in distant adipocytes [34]. Antioxidant and blood glucose-lowering chemicals found in *Vigna unguiculata* L. (cowpea) have aided patients. Over the course of 20 h, researchers delivered extremely high dosages of cowpea peptides (0.1, 1, 10, and 100 ng) and insulin (100 nM) to L6 skeletal muscle cells. A Western blot analysis of proteins from treated cells is also being utilised to determine whether or not Akt activation has occurred (a form of protein kinase B; PKB). Cowpea peptides can phosphorylate Akt during cell implantation, consistent with the findings of the study. Cowpea peptides can stimulate insulin signalling in skeletal muscle cells, which is consistent with previous research. Cowpea peptides can act as a substitute for insulin by duplicating its signalling function [77].

The article "A Treatment to Cure Diabetes Using Plant-Based Drug Discovery" was published in 2022. Journal: Evid Based Complement Alternat Med.

Peptides synthesised as seed peptides from *Linum usitatissimum* (flax) protein hydrolysate (50 kD) outperform L6 mobile glucose uptake [78]. Arrived: peptide fraction from *Momordica charantia* L. Hypoglycemia is most likely diagnosed by an in-person or in-female examination. The MC2-1-five fraction lowers blood glucose levels with a useable resource of 61.70% and 69% of the total population, respectively. Alloxan-treated diabetic rats lost 18% of their bodyweight in just 4 h [79]. For a minute, examine the protein in *Momordica charantia* L. pulp. Insulin secretion and glucose levels were both reduced in C2C12 and 3T3L adipocytes when a protein derived from pulp was supplied to the cells, in accordance with an in vivo examination [80], [81]. Insulin uptake and clearance are improved in diabetic mice, thanks to the useful resource of in vitro digestion of the plant-derived insulin receptor binding protein (mcIRBP), which has 68 residues, to provide mcIRBP-19, which increases insulin receptor binding and activates PDK1, Akt, and the expression of glucose transporter 4, McIRBP-19 [40]. *Momordica cymbalaria* L. fruit's 17 kD protein, Mcy protein, has been studied in vivo for its hypoglycemic effects [82]. It was further confirmed that the peptide fraction improved glucose absorption in muscle cells by activating AMK, a cellular enzyme [83].

Researchers discovered that when they were given a protein extract produced from the Cucurbitaceae family of seeds, which includes *Telfairia occidentalis* Hook.f., *Citrullus lanatus* L., *Lagenaria siceraria* Molina, and *Cucurbita moschata* Duchesne, their blood sugar levels plummeted dramatically [84]. A peptide isolated from *Bauhinia variegata* L. leaves mimics insulin in terms of immunological reactivity and in vivo detection [85]. Studies on *Zea mays* L. (Zein) seed protein hydrolysate in GLUTag cellular lines revealed that it increased the synthesis of the hormone GLP-1 in rats' ileum and duodenum [86]. Glycine supplements the production of p-IR, p-IRS1, and the membrane-GLUT4 protein to reverse the hypoglycemia effects of diabetic mice on C2C12 cells. In C2C12 ells, glycine improves glucose absorption [87]. Soymorphine-5, also known as opioid, reduces blood glucose levels in diabetic KK-Ay mice through activating the adiponectin and PPAR systems [88]. Insulin sensitivity has improved, and metabolic issues have been addressed with the help of rice bran protein hydrolysate [89]. To isolate the protein, the fruit pulp of the *Momordica dioica* Roxb fruit was employed. Even when taken in its diabetic form, this medication lowers diabetics' blood glucose levels [90]. Peptides similar to insulin or peptides meant to imitate insulin are also thought to be present in the blooms of extraordinarily excellent plants by a variety of plant scientists [91].

The article "A Treatment to Cure Diabetes Using Plant-Based Drug Discovery" was published in 2022. Journal: Evid Based Complement Alternat Med.

### 1.7. Overcoming Obstacles with Peptide Drugs

Success and popularity are directly linked to how quickly and easily a treatment may be implemented [64]. As the vast majority of medicines on the market today are taken orally, oral medication substitution is the most well-known and widely used technique [92]. The stomach's environment can be experienced by bypassing the gastrointestinal membrane with energetic tablets taken orally. Small molecules, in contrast to large macromolecules that dissolve in the gastrointestinal system and cannot be permeable in their intact form to collect a specific cause without degradation, can remain on the stomach pH and bypass the barrier [92]. As the medical period progresses, an increasing number of peptide drug therapies are being examined for their restoration potential in the treatment of a wide variety of ailments [93]. There has been a longstanding problem with oral bioavailability of peptide-based totally medications despite the fact that their genuine goal, usefulness, and effectiveness are accurate. Peptide medications have a high rate of side effects, which is a major downside [62]. Recombinant peptide synthesis is a method by which biotechnology's successes can be achieved at lower costs and with less strength. Bioactive peptides derived from natural resources are gaining commercial interest, but large-scale production has been hampered due to lack of adequate generating methods [94].

The half-lives of peptide-based therapy pills are often only a few hours long, which is a source of concern. Peptides are broken down into amino acids by stomach acid and blood peptidases, which are quickly eliminated from the body and cause a decrease in the peptide half-life. It is imperative that peptides be adjusted to be more long-lasting and less hazardous because of their half-lives. More and more importance are being placed on nondegradable polymers and polymeric matrix as peptide treatments adorn, with a reduction in the famed dose timetable being taken into account [95]. Enzymes can be used to replace amino acids that are prone to cleavage, which further improves the peptide's half-lifestyles [7]. Peptide oral delivery has been tested in the past, but its application is limited due to the fact that the GI system breaks down peptides [96]. Novo Nordisk has developed an oral version of semaglutide in the early stages of clinical studies. Oral medication delivery has one of the main downsides, which can be mitigated by the employment of noninvasive methods such as nasal and pulmonary channels that give recuperation and healing strategies to the circulation immediately [97].

The article "A Treatment to Cure Diabetes Using Plant-Based Drug Discovery" was published in 2022. Journal: Evid Based Complement Alternat Med.

### 1.8. The Destiny of Peptide-Based Totally Therapeutics Is Brilliant

Therapeutic peptides are becoming increasingly popular because of the fact that peptides are more strong, selective, and easy to use than small compounds. There is a good chance that this trend will continue in the future [98, 99]. Researchers and pharmaceutical companies can use ordinary synthesis and drug format approaches to multiply peptide-based totally in reality therapeutic possibilities. Using a recombinant protein from bacteria, yeast, or fungi, a desired peptide can be synthesised [100]. Artificial peptide synthesis has progressed to the point where it can mimic the effects of natural peptides without relying on animal delivery. One of the advantages of peptides that can be drug-conjugated is that they have several functionalities [98]. There is a risk of peptide breakdown when being fed on, despite the fact that the most convenient form of delivery is peptides. The most common method is intravenous peptide manipulation; however, new studies are being conducted in this area. Attempts have also been made to give the drug orally and transdermally via intranasal administration. Peptides may be used to aid in the diagnosis of disease due to their attractiveness as symptoms. Vaccines can also benefit from the use of peptides, as has long been shown [95, 101].

Researchers employed the same techniques shown in Figure 4 [94] to isolate and characterise plant peptides. The combination of X-ray crystallography and nuclear magnetic resonance (NMR) has greatly assisted herbal peptides (Figure 3). Natural peptide shapes have benefited greatly from advances in X-ray crystallography and nuclear magnetic resonance (NMR) [102].

Characterization techniques such as electron microscopy, fluorescence resonance energy transfer, and chemical flow-linking have advanced in the previous year [103], [104]. Peptide combinations can be thoroughly investigated using mass spectrometry, which finds the best possible form for each and every one. There are numerous approaches for mass spectrometry-based amino acid sequencing, including facet pinnacle-down and bottom-up. The molecular weight can be estimated in pinnacle-down sequencing without hydrolysis by using the intact protein fragmentation pattern. Down-top sequencing, in which proteolytic digestion is completed prior to MS analysis, is a frequent approach. Protein identification software application is available, and it is based entirely on the amino acid collection's criteria [105].

The article "A Treatment to Cure Diabetes Using Plant-Based Drug Discovery" was published in 2022. Journal: Evid Based Complement Alternat Med.

## 2. Discussion

Plants, on the other hand, are an excellent resource for cultivating an entirely unique therapeutic candidate. A small fraction of the most well-known drugs and lead will be used. In the meantime, plants are being studied for the production of proteins and bioactive peptides for the treatment of ailments, since the focus of study has shifted from small molecules to biomolecules due to numerous advantages. Plant hormones have long been thought to be the most ultramodern way for cells to communicate, despite the fact that plant proteins and their homes have just recently begun to be seen. As our understanding of those signalling pathways expands, a variety of secreted peptides and short RNAs are being proposed as means to control cellular communication by changing molecular structure. After gastrointestinal digestion, proteins can be transformed into bioactive peptides with a greater tissue affinity for a specific receptor. Several recent studies have emphasised plant proteins and their bioactive peptides as a potential competitor in the treatment of a number of illnesses, particularly metabolic and lifestyle-related illnesses such as cancer, diabetes, and weight problems. A cutting-edge methodology and technical leap forward allows for the clean isolation, purification, and characterization of proteins and peptides in a short amount of time, reducing the overall length of the invention process.

The bulk of bioactive peptides used to treat diabetes appears to have come from synthetic or recombinant production, and each of them is most likely included in the drug's daily dosage. Plant-based biomolecules may be necessary to make peptide therapy more cost-effective. This research is based on bioactive peptides extracted from a number of plant components, including leaves and seeds, and stop results. Although bioactive peptides can be found in leaves, pulps, and entire preventive outcomes, seeds are thought to provide the greatest bioactive peptides to the general public.

Protein hydrolysate derived from plant aqueous extracts has been shown to disrupt the enzymes and transporter systems that cause diabetes, through in vitro and in vivo experiments. An exciting journey into the molecular structures and mechanisms of action of plant-based totally bioactive peptides is required, as well as a fantastic method for using those bioactive peptides as a capability restoration option.

The article "A Treatment to Cure Diabetes Using Plant-Based Drug Discovery" was published in 2022. Journal: Evid Based Complement Alternat Med.

## 3. Conclusion

Treatments for type 2 diabetes based mostly on artificial pharmaceutical capsules have been proved in epidemiological studies to cause minor to extreme terrible facet consequences. It is believed that the bioactive peptides derived from flowers inhibit alpha-glucosidase, alpha-amylase, DPP-IV, and glucose transporter systems. A plant peptide fraction has been examined in vivo and positioned to have insulin-mimicking homes in animals. Plant-derived bioactive peptides are underutilised in assessment of unique herbal product lessons. Peptides from plant reminiscence cannot be recognized, purified, and studied because there are not any good enough instrumental strategies. This can be an extremely good time to start strolling with the plant peptides of your choice, way to modern advancements in LCMS, LC-NMR, and X-ray crystallography. In the future, plant peptide studies must benefit from the systematic test that involves dereplication for early peptide identification, goal identity, and in vivo trying out.

## Figures and Tables

**Figure 1:** Diabetic discovering from various disorders [12] (Statement Note: In the figure legend reproduced from Patil S.P., Goswami A., Kalia K et al.' Plant-Derived Bioactive Peptides: A Treatment to Cure Diabetes. Int J Pept Res Ther 26, 955–968 (2020). https://doi.org/10.1007/s10989-019-09899-z).

**Figure 2:** Population wise country report of diabetics [19].

**Figure 3:** Proposed structure of bioactive peptides [40].

**Figure 4:** Plant peptides being isolated, purified, and characterised in accordance with current best practises [94].

**Table 1:** Types of diabetics and its methods [20].

Type	Method
Type 1 diabetic (juvenile)	Decreased insulin
Type 2 diabetic	Glucose storing cells developing insulin resistance
Type 3 gestational diabetes	Increased danger of health issues
Type 4 other diabetes	For pregnancy women

**Table 2:** Plants possessing antibioactivity for diabetics [20].

S. no.	Plants	Used sequence
1	Babul	Sore throat
2	Aloe vera	Changes in urine colour and vomiting are among the side effects that can accompany bulimia.
3	Garlic	Immune system booster; reduces hypertension; antibacterial and antifungal qualities
4	Beetroot	Improve the condition of hypertension
5	Neem	Pain, fever, and infection are all symptoms of infection.
6	Church steeples	Cultural porphyria is a skin ailment.

**Table 3:** Hydrolysate from plants for antidiabetic activity [40].

S. no.	Plants	Part	Activities
1	Araliaceae	Roots	Different hypoglycemic and insulin substances, as well as glycans such as panaxan A through P and ginsenoside Rb1, have been identified from the roots of diverse plants. Antilipolytic properties have been attributed to a number of substances.
2	Rhodophyta	Leaf	C was found to contain two distinct polypeptide fractions.
3	Cucurbitaceae	Fruits and seeds	*Momordica charantia* was used to produce p-insulin, which was extracted from the fruit, seeds, and tissue (bitter gourd)
4	Leguminosae	Seeds	The protein *A*. *melanoxylon* and *B. retusa*, which was isolated from seeds, was investigated.
5	Fenzl	Fruits and seeds	*Momordica cymbalaria* significantly reduced fasting plasma glucose levels in diabetic mice caused by streptozotocin.
6	*Coix lacryma-jobi* L. var. ma-yuen Stapf.	Grains	Adlay grains have a significant amount of prolamin, which is an alcohol-soluble protein belonging to the prolamin group.
7	*Oryza sativa*	Rice bran	Insulin resistance was improved by consuming a functional meal.

The article "A Treatment to Cure Diabetes Using Plant-Based Drug Discovery" was published in 2022. Journal: Evid Based Complement Alternat Med.

## Data Availability

The data used to support this study are included within the article and are available from the corresponding author upon request.
